# Psychometric Model of College Students Based on Time Series Analysis and Its Application in Educational Management

**DOI:** 10.1155/2022/9550463

**Published:** 2022-05-06

**Authors:** Lu Lu

**Affiliations:** Guangdong Nanhua Vocational College of Industry and Commerce, Guangdong Guangzhou 510507, China

## Abstract

The psychological measurement method of college students is a hot issue in the field of educational management research. Based on the time series analysis theory, this paper constructs a psychological measurement model for college students. This paper analyzes the psychometric behavior data, uses the time series analysis method for behavior prediction, deeply mines the relevant component information of the psychometric data, and solves the problems of weak correlation between the functions of the psychometric platform and low data accuracy of the psychometric model. At the same time, taking the intervention target group and the intervention mode as the basic variables of the intervention classification system, combining these two dimensions, a two-dimensional classification framework for psychometric intervention was proposed, and four types of different psychometric intervention measures were applied. During the simulation process, a psychometric trajectory matrix was constructed, and a two-dimensional data extraction network was used to extract the psychometric pattern data of a certain period of time. The experimental results show that using the student mental state data as a label can obtain a low-coupling training set classification for psychometric effects of college students.

## 1. Introduction

With the development of the Internet and information technology, people's psychological measurement life has been accelerated, new ways of thinking and cognition have been provided, and psychological measurement has gradually been recognized by the public [1]. This brand-new psychometric and educational model will surely further drive the implementation and reform of educational informatization. The vigorous development of psychometrics is also accompanied by many challenges. Due to the solidification of students' psychometric thinking, psychometric platforms are not valued; teachers only use psychometric platforms to complete related tasks and do not devote energy to psychometric-related knowledge. Insufficient functions of the measurement platform and slow maintenance lead to poor psychological measurement experience for psychometric users [2–4]. Among the many challenges in the psychometric platform, the rapid loss of psychometrics and the low rate of course completion are the most frequent and prominent consistent phenomena and analyze predictions to find their crux. The analysis of the existing behavior prediction research shows that there are problems such as timeliness lag, too simple prediction methods, unprofessional prediction models, and low accuracy [5–8].

Models about psychometric outcomes are used to explain related psychometric concepts. The model established by Yan [9] specifically interprets the results of psychometrics, including seven types: participation of psychometrics, effectiveness of technology, cognitive participation, self-efficacy, psychometrics, intuitive attitude, and psychometric superiority. Through this study, Martínez et al. [10] deeply analyzed the specific influencing factors that lead to changes in psychometric results and summarized these factors into four categories: psychometric characteristics, teacher characteristics, curriculum-specific characteristics, and technology-related characteristics. Won and Shirley [11] verified the actual effect of each factor on psychometric results. According to the subject of intervention, intervention can be divided into human intervention and automatic intervention. Manual intervention is mainly used in traditional classroom teaching. After teachers find problems, they directly participate in the teaching intervention of psychometrics, such as adding exercises, dialogues, adjusting teaching methods, and psychometric activities. Automatic intervention mainly refers to informal psychometric or mixed psychometric activities. Technically supported interventions in measurement such as personalized psychometric systems or interventions implemented by adaptive psychometric systems. Teachers use equipment psychometric mobile terminals to conduct psychometric interventions [12–16]. These methods are individualized structured, individualized unstructured, collective structured, and collectively unstructured. In addition, some researchers have proposed different intervention mechanisms for teacher-led and student-autonomous psychometric measures.

This paper mainly adopts the literature analysis method and mathematical statistics research method and mainly focuses on the following contents. The first is to sort out the domestic and foreign literature on the current research status through the literature analysis method and determine the development status of the research in this field, which lays a theoretical foundation for the research problem. Secondly, according to the three-dimensional time series psychometric behavior classification model proposed in doctoral dissertation, as well as summarizing the related researches on psychometric behavior, combined with the characteristics of the psychometric platform in this paper, a psychometric behavior classification model is constructed. Third, based on the psychometric behavior data in the psychometric platform, from the perspective of a time series classification model, this study uses statistical knowledge to predict psychometric behavior. In order to further optimize the recognition effect of the model, this paper proposes a mental health problem recognition algorithm based on the time series analysis model. The online trajectory matrix is constructed, the two-dimensional convolutional neural network (2D-CNN) is used to extract the online mode of one day, the memory network is used to capture the time dependence between each day, and the depth psychological measurement is designed by combining the basic features and the online trajectory mode. Experiments show that precision reaches 0.71, recall reaches 0.75, and *F*1 measure reaches 0.72, which can identify 75% of students with mental health problems.

## 2. Methods

### 2.1. Time Series Dimension Analysis

In the ideal time series case, *h*1(*t*) is an eigenmode function component. But in fact, it also needs to repeat the above process until the conditions of the time series are satisfied, thereby decomposing the first time series component *c*1(*t*) = *h* − *k*(*t*), which represents the highest frequency component of *x*(*t*). In this process, the removal of the superimposed wave makes the instantaneous frequency meaningful; at the same time, since the adjacent waveforms are also smoothed, resulting in the removal of meaningful amplitude fluctuations, the conditions for stopping this process are the number of poles and zero crossings, the point difference is at most 1, and the upper and lower envelopes are locally symmetrical about the time axis. By obtaining *c*1(*t*), then *r*1(*t*) = *x*(*t*) − *c*1(*t*), until the stopping condition is satisfied; finally, the original signal is decomposed into *n* time series and a residual *rn*. The decomposition process is empirical, adaptive, and based on the local features of digital signals [17–19].

(1) $$\begin{array}{c} c\left(w,w^{\prime }-t\right)=\int \frac{-t+\sqrt{t^{2}-4tc}}{2tx}dx-\int \frac{-w+\sqrt{t^{2}-4tw}}{2tw}dw. \end{array}$$

In the process of time series data preprocessing, for consumption data, since consumption records, student information, and store information are stored in three tables, we will connect them. For the web log data, due to the large amount of noise data in the data, it is necessary to remove the noise data according to the request URL; at the same time, because there are too many types of URLs in web logs, we unified them into seven categories. For grade data, there are a large number of missing values, and it is necessary to find out the calculation formula according to the law of existing values and fill in the missing values. Taking the random correlation matrix ruler as the null hypothesis, comparing the statistical characteristics of the correlation matrix of college students' psychometric data in Figure 1 with the statistical characteristics of the random correlation matrix ruler, the characteristics of the correlation matrix of college students' psychological measurement data can be obtained, which can be used for emotional physiological measurement data. The correlation of signal time series is studied [20–23].

The essence of time series processing of college students' psychometric data is that the energy of signals containing noise is generally concentrated in low frequency and short, and the higher the height, the less energy. Therefore, there must be a time series component so that in the following components the signal energy is less, which is the dominant mode, and its previous components are heavy, and the noise is the dominant mode, and the purpose is to find this time series. The process of decomposing the time series into several components from low to high reflects the characteristics of self-adaptation. According to the prediction value of the current base classifier and the loss value of the actual value as the target of the latter base classifier, the establishment of the latter base classifier is to reduce the loss generated by the former base classifier. The method of reducing the loss is to let the former base classifier. The residual of the weak classifier is reduced in the direction of the gradient, and then, multiple weak classifiers are accumulated to obtain a strong classifier.

### 2.2. Psychometric Training Data

According to the research results of psychometric behavior classification, the classification model is suitable for analyzing related psychometric behaviors in online platforms. Behavior within the platform is further segmented using a network behavior time series classification model. As mentioned above, it constructed a three-dimensional psychometric behavior time series model, which can be very comprehensive and specific to classify psychometric behaviors from multiple aspects and dimensions. Among them, the first two lines of dictionaries represent two dictionaries, respectively, and each picture is regarded as the feature base vector representation of a frame, that is, it is assumed that there are five feature base vectors each. It is the input data, and each image is equivalent to one frame of feature vector, that is, three frames of data are intercepted from the input. They are the coefficients obtained by traditional sparse coding algorithms.

(2) $$\begin{array}{c} \left|f\left(w-t,w^{\prime }-t\right)\right|=\sqrt{t^{2}-t+1}+\sqrt{t^{2}-t}+\sqrt{t^{2}-t-1}+\cdots +\sqrt{t^{2}-t+n}. \end{array}$$

Therefore, according to the network behavior model, the experiment classifies various psychometric behaviors in the database according to the three dimensions of structure (S), function (F), and mode (F) to reveal the psychology of the platform's psychometrics in measurement characteristics. This article will use the time series psychometric behavior model to organize and summarize various network behaviors in the platform. However, in order for the model to be more suitable for the classification of specific psychometric behaviors in the psychometric platform, the time series model also needs to be adjusted and adjusted according to the actual situation of the psychometric platform in which it is used.

As can be seen from the figure, without considering the time sequence, when the input data is similar to the feature base vector pose in the dictionary, the result as shown in paper will be obtained, but such a result will cause interference and misjudgment. In order to solve the above problem, there should be a regular term that can make the coefficient vector reflect the time order of the input data vector and suppress the time series error. This is equivalent to ensuring normal coefficient vector output when the time order of the input data vector is the same as that expressed by the base feature vector of the subdictionary in the dictionary, when the time order of the input data vector is the same as the base feature of the subdictionary in the dictionary. When the time sequence of the vector expressions is not the same, the blindly increasing coefficient value in the coefficient vector is suppressed.

The quality of the model performance cannot be seen intuitively, and it needs to be measured by the evaluation indicators in Figure 2. Confusion matrix is an index to evaluate the performance of the model; it is mainly used to judge the performance of the classifier. The confusion matrix has four basic elements, which are True Positive (TP), False Negative (FN), False Positive (FP), and True Negative (TN). Below we will introduce the specific meanings of these four elements in detail. TP: the number of students who are predicted to be positive samples and the real marks are also positive samples, that is, the number of students who are predicted to have psychological problems and that the student does have psychological problems. FN: it is predicted as a negative sample, and it is actually marked as a positive sample, that is, it is predicted that there is no psychological problem, but the student has a psychological problem. FP: it is predicted as a positive sample, and it is actually marked as a negative sample, that is, it is predicted to have psychological problems, but the student does not have the number of psychological problems. TN: the number of predicted negative samples, and the real marks are also negative samples, that is, the number of students who are predicted to have no psychological problems, and the student does not have psychological problems.

### 2.3. Sequence Encoding and Acquisition

In order to calculate the deviation between the psychological measurement data of college students and the prediction of random matrix theory, it is necessary to first assume a set of uncorrelated normalized time series of length *D*, where the values of *D* and IV are the same as the time series of emotional and physiological signals. The length and the number are the same. Four uncorrelated normalized time series of length *D* are composed of *N* × *T*-dimensional data matrix *A*, and the correlation matrix of the data matrix is constructed. For the decomposed time series, the low-frequency time series is removed to preserve the high-frequency time series, the high-frequency time series is removed to preserve the low-frequency time series, the high-frequency and low-frequency time series are removed to preserve the intermediate time series, and the intermediate time series is removed to preserve the high-frequency and several combinations of low-frequency time series, respectively, forming high-pass, low-pass, band-pass, and band-stop filters. The advantage is that it can preserve the nonlinearity and nonstationarity of the signal to the greatest extent, and there is also the possibility that the energy of the signal may be lost in the process of discarding the time series, and the data of discarding the time series depends entirely on prior knowledge.

(3) $$\begin{array}{c} \overset{u=1}{\underset{u,v}{\sum }}g\left(u\left(t\right),v\left(t\right)\right)\times g^{-1}\left(u\left(t-1\right),v\left(t-1\right)\right)=\overset{u=1}{\underset{u,v}{\sum }}\frac{u\left(g\left(t\right),g\left(t\right)\right)}{v^{-1}\left(g\left(t-1\right),g\left(t-1\right)\right)}. \end{array}$$

After unifying the grade data, we also observed that there are missing values in the grade point column in the student's historical grade table. Since GPA is the result of multiplying GPA and course credits, missing GPA will result in missing corresponding GPA. By observing the existing grade points, we found out the calculation rules of grade points, as shown in Table 1, in which the corresponding relationship between the calculated grades and grade points is shown in the text. Next, according to the formula, we can calculate the missing grade point.

For college students, the biggest pressure on grades is to fail a course. Failure to pass the makeup examination and retake will affect their smooth graduation. For the undergraduates of our school, failing a subject may cause them to repeat the grade. Referring to the relevant regulations of the undergraduate student handbook, the college will count the failing grades of the undergraduates of each grade after the end of each semester. If a student's failing grade exceeds 25 points (including 25), the student will enter the probationary stage in the next semester, that is, in the status of repeating grades. After completing the required credits during the probationary period, they can follow the students of the next grade for psychological measurement; if they fail to complete the required credits, they will be forcibly withdrawn from the school. Therefore, failing grades is the best feature to reflect the pressure of grades. The method of counting the passing credits is traverse the student's historical score table; if the credit acquisition method (QDFS) value is makeup examination, the corresponding credits will be counted as passing credits.

### 2.4. Dynamic Programming of Measurement Scales

The article obtains the student's mental state table; each record in the table contains the student's student number, gender, department, grade, class, attention level, and update time, as shown in the text. The level of concern includes three levels: light, medium, and severe. “Light” indicates mild mental health problems; “medium” indicates moderate mental health problems; “severe” indicates severe mental health problems. In this paper, our target is a binary classification problem, that is, students with mental health problems and normal students.

Therefore, if the expression order of the input matrix and the eigenvectors of the subdictionary are the same in time, an optimal and limit expression of the subcoefficient matrix *j* should be in the form of a positive diagonal matrix, that is, except for the coefficients on the diagonal position has a value and zero elsewhere. If the expression order of the input matrix and the eigenvectors of the subdictionary are inconsistent in time and if the behaviors are mutually inverse, the optimal and limit expression is that the coefficient values are all zero. Such coefficient expressions can completely distinguish and identify different classes of behavior.

(4) $$\begin{array}{c} K\left(x,y\right)-\text{scanner}\left(x,y\right)=\left[\begin{array}{cc} k-\text{scan}\left(x,y\right) & k\left(x\right)-\text{scan}\left(y,x\right)\\ k\left(y\right)-\text{scan}\left(x,y\right) & k-\text{scan}\left(y,x\right) \end{array}\right]. \end{array}$$

For the requested URL is an IP address, we directly remove such records. For the useless records generated by loaded web pages containing static resources, we exclude static resources based on resource extensions. The URL requested by the user usually contains the name of the resource. These names are composed of the file name and the file extension. The type of the file can be known according to the file extension. For example, js means JavaScript script, jpg means image, and html means hypertext. We have made statistics on common static resources. When traversing each file, we judge whether the extension of the requested resource belongs to static resources, and if so, remove this record. For the third question, according to the properties of the website, URLs can be divided into different types, and the URL type can indicate the purpose of the user visiting the website. In this paper, we choose n-gram-based URL classification because it has a large trade-off between computational complexity and accuracy.

## 3. Results

### 3.1. Sequence Threshold Classification

Among the 4295 pieces of data selected, some data are operational data of teachers and network teaching administrators, in order to ensure the accuracy and rigor of the research. The researchers eliminated the behavioral data generated by teachers and teaching managers in the 4295 pieces of data, and the remaining 3282 pieces of behavioral data were the psychometric behavioral data used in this study. First of all, in order to draw the overall sequence diagram of psychometric behavior, read the behavior data file and load the various packages required for drawing and draw.

The correlation matrix was constructed for the 8 channels of physiological signals collected, respectively. Because the psychological measurement of college students is reflected in the variation law of physiological signals in Table 2, adding a bias to the overall sampling and recording sequence of each signal does not affect the analysis of the variation rule of physiological signals, while the additional bias can make all physiological signal sequences a positive value. It can be seen that the number of frames (that is, the number of column vectors) of the subdictionary is equal to the number of column vector elements of the subcoefficient matrix *j*, and the number of column vectors of the subcoefficient matrix *j* is equal to the number of frames of the input matrix.

It can be seen that the smaller the entropy value of a behavior is, the more concentrated its probability distribution is with the time interval, and the higher its regularity is. However, we found that if one student only occasionally went to the cafeteria to eat during the concentrated time period and another student often went to the cafeteria to eat during the centralized time period, although the regularity of the two students going to the cafeteria was different, they will also be similar entropy values.

### 3.2. Normalization of Population Factors

The first step of normalization is because the behavior data experiment stores the collected network behavior data in excel software. In order to read the data in R, the readxl package is used for data entry, and the time series analysis of the data is required, so the forecast package is the so-called forecast package for forecasting. The tidyverse package is a summary package. The various packages included are mainly to help with drawing, so we use these three packages for analysis, forecasting, and drawing. We used the ggplot package to plot the aggregated network behavior data, resulting in a time series diagram of the psychometric platform as a whole as shown. The purpose of this paper is to make use of this temporal information, treat the entire input as an overall multidimensional time series, and strengthen their inherent temporal information. The sparse coding method based on each frame alone cannot represent the underlying temporal information between frames, so better methods are needed to express it. The method described below in this paper is to enable the represented sparse coefficients to reflect temporal information and to preserve the temporal order between the feature vectors before encoding.

According to the prior knowledge, the maximum MAXLEN and minimum MINLEN lengths of the subsequences are set, the information gain is measured for each subsequence in the dataset in Figure 3, and the shapelet with the largest information gain is selected as the basis for constructing the classifier. In the process of calculating the information gain of a subsequence, the distance between the subsequence and all the time series in the dataset needs to be calculated, so there is a dividing point dt as the distance threshold. According to the distance between the subsequence and the time series in the dataset, the datasets are divided into two categories. Then, by calculating the information gain of each division point dt that may divide the time series into two categories, take the maximum value as the information gain of the current subsequence, compare it with the information gain of other subsequences, and take out the largest information gain in all subsequences.

### 3.3. Feature Extraction of Network Data

The data feature extraction obtains the time series adaptive college students' psychometric data, uses wavelet transform to extract its high-frequency signals, time series extracts its low-frequency signals, and inputs them into the adaptive filter as noise, so as to process college students' psychometric data, improving the signal-to-noise ratio of college students' psychometric data, laying a solid foundation for better extraction of effective features in the next step. Aiming at the lack of prior knowledge of college students' psychometric data, combined with the time series characteristics of college students' psychometric data, a local feature descriptor of college students' psychometric data is constructed based on the time series shapelet recursively and recursively. The characteristic sequence of the data is extracted, and the characteristic information of different media contained in the psychological measurement data of college students is effectively extracted.

On the basis of the existing 6 types of discrete emotion sample library, in order to verify the model selection and model prediction and recognition ability, the sample set in Figure 4 needs to be redivided. The scale of each emotion class sample library is happiness, surprise, disgust, sadness, anger, and fear with 216, 167, 100, 235, 349, and 217 samples, respectively. Divide the various sample libraries into three parts: randomly select 1/3 of them to form dataset I for classifier training; and randomly select 1/3 to form dataset II for feature selection and the rest constitute dataset III for validation of the model's predictive ability. In order to prevent the overfitting of the system model to the fixed dataset and enhance the generalization ability of the model, the random construction process of the above dataset was repeated 50 times, and the prediction ability of the model used the average hit rate TPR and false alarm rate of 50 cross-validation FPR as a measure.

## 4. Discussion

### 4.1. Nearest Neighbor Analysis of Time Series Data

The stationarization test is carried out separately for the overall psychometric behavior time series data. According to the processed psychometric behavior time series diagram, it can be clearly found that the fluctuation of the data is very huge. Therefore, in order to establish a prediction model, it is necessary to stabilize the time series. Here, we choose the logarithmic method and then perform the unit root test on it to ensure that the processed data is a stationary time series. Sparse representation provides a good encoding method for behavior recognition data features. The usual method is to first decompose the input sequence into frame-by-frame data, that is, the feature vector at each moment, and then encode each frame of data independently, and finally encode it. The coefficient vectors corresponding to each frame of data are put together. But such methods ignore the strong temporal correlation between frames.

(5) $$\begin{array}{c} \left\{\begin{array}{c} \beta \left(a,b\right)=\eta \left|a\left(t\right)\right|-\eta \left|b\left(t\right)\right|,\\ \alpha \left(a,b\right)=\lambda \left|a\left(t\right)\right|+\lambda \left|b\left(t\right)\right|. \end{array}\right. \end{array}$$

The time scale of constructing a time series of length *r* from the signal sequence is *t* = 8 seconds. At this time, the *Q* value is close to the lower limit value of 1. The time series reflects the slow changing law of the signal. The analysis of the time series correlation matrix shows that the time-accumulated physiological response of emotion, that is, the duration or required reaction time for emotional and psychological experience to be reflected in the changing laws of physiological signals. When the number of data samples is constant, a larger value of *Q* corresponds to a smaller time scale. When *f* is small enough to reflect the transient law of the signal, the properties of the signal time series correlation matrix constructed from this can reflect the instantaneous emotional state. Since skin conductance and heart rate are ultralow-frequency slowly varying signals, take the time scale *At* = 0 for them and 5 seconds to show its transient law.

Here, we use the tseries package in the R language and use the time series test in this package. The null hypothesis of the test is that “the original sequence has a unit root,” that is, the overall psychometric behavior time series data is not stationary. It can be found from the results that the *P* value is equal to 0.01, and then, the null hypothesis is rejected, that is, the data after taking the logarithm is stationary. In the same way, the three categories of psychometric behavior data under the *F* dimension are tested for stationary time series, and it is found that the *P* values are all less than 0.05, so the above four time series are all stationary time series.

### 4.2. Psychometric Model Simulation Implementation

In order to establish a more accurate prediction model, the key link is to order the model. There are three main methods of order determination at this stage: the order determination method based on the autocorrelation function and the partial correlation function, the determination of the order based on the F test, and the use of the information criterion to determine the order (AIC criterion and BIC criterion). The model is ordered based on the method of autocorrelation function and partial correlation function. The dictionary is divided into multiple groups of subdictionaries, each group of subdictionaries includes multiple feature base vectors (column vectors), and the dimension of the column vector is also the feature dimension. According to the grouping of the dictionary, the sparse coefficient matrix is a group of subcoefficient vectors of the same color and corresponds to the input vector and the subdictionary. The number of column vectors is the same as the number of column vectors of the input matrix column vector dimension. The number is the same as the number of base eigenvectors (that is, the number of column vectors) of the dictionary.

It can be seen that the value of the autocorrelation coefficient decreases slowly, so it is tailing, and the value of the partial autocorrelation coefficient in Figure 5 is still outside the critical range (the range inside the dotted line in the figure) in the later periods, so it does not belong to the tailing. Therefore, the PACF graph is also tailing, so we choose the ARMA model for modeling. The parameter of AR(1) model is 0.4641, the parameter of MA(1) is -0.0969, the constant term of autocorrelation is intercept = 3.0125, and the constant term of partial autocorrelation is 0.1510. According to the AIC information criterion value, the good fitting of the model is judged. The AIC value of the bad ARIMA(1,0,1) model is equal to 352.49, indicating that the fit of the model is not bad.

### 4.3. Case Discussion and Analysis

In the example, it can be found that the generalized variance, Ljung-Box test detection and ACF value of residual error, GVTEST value and LBQ value, the null hypothesis of these two tests is that the sequence is a random sequence; it can be found that most of the *P* values of the Ljung-Box graph are all greater than 0.05, so the data in these time series are random data, and the data in a small number of lag periods are less than 0.05, so the null hypothesis is rejected; then, the data in the series has a relationship with the data in these lag periods, indicating that in the it. The individual values may not be independent and random during this time. On the whole, most of the data in the lag period conform to the null hypothesis that the sequence is a random sequence, which means that the residual test of the model is not bad. The model is used to predict and fit as shown in the text. It is found that the predicted time series is consistent with the actual time series trend, indicating that the overall psychometric behavior prediction model established by it is better.

Then, the distribution of the eigenvectors of the correlation matrix *C* is counted and compared with the distribution of the eigenvectors of the random matrix scale. The comparison is carried out from two aspects: (1) the eigenvector *U* corresponding to the maximum eigenvalue of the correlation matrix of the emotional physiological signal sequence outside the theoretically predicted maximum eigenvalue and (2) the steps of the eigenvectors corresponding to the eigenvalues of the correlation matrix of the emotional physiological signal sequence within the range of the theoretically predicted eigenvalues.

In the research process of college students' psychometric data, firstly, the data processing methods of several existing college students' psychometric data are deeply studied and then combined with the time series data mining method, and the medium information characteristics in college students' psychometric data are analyzed. It is extracted and analyzed, and finally, the psychological measurement data of college students are classified according to the characteristics extracted by the analysis, and the processing and analysis results are presented through visual effects.

## 5. Conclusion

Through the research on the existing college students' psychological measurement data processing and analysis methods, this paper improves the existing college students' psychological measurement data processing technology, uses time series analysis to improve the signal-to-noise ratio of the data, and unifies the center point and scales the coordinate data. The transformation of unification and angle unification makes the coordinate features have scale invariance and rotation invariance, and the experimental analysis also confirms that it has better robustness. According to the psychological measurement principle of college students, the psychological measurement data of college students comes from the real-time sampling process that occurs at equal intervals of sampling pulses and has the characteristics of time series. During the experiment, the sparse representation algorithm of time series analysis was used as a multidimensional time series modeling method, multidimensional analysis of time series was carried out, and a regular term added to supervise time series chaos was used to suppress errors in motion time so that traditional sparse coding could be processed with a multidimensional time series modeling approach with motion information. The important influence of time series information on sparse coefficients and the improvement of classification accuracy are verified through experiments.

## Figures and Tables

**Figure 1:** Time series dimension topology.

**Figure 2:** Classification and comparison of psychometric training data.

**Figure 3:** Time series sample population factor normalization.

**Figure 4:** Feature extraction distribution of time series network data.

**Figure 5:** Psychometric model information criterion legal order distribution.

**Table 1:** Time series coding.

	Group series	Model first point	Model final point	Model average point
Grade table 1	Grade a	60.557	43.701	52.129
	Grade b	46.237	11.765	29.001
	Grade c	52.648	32.078	42.363
Grade table 2	Link a	2.258	48.341	25.300
	Link b	76.900	39.401	58.151
	Link c	10.942	46.608	28.775
Grade table 3	Course a	48.93058	44.53739	46.73399
	Course b	42.90767	28.23115	35.56941
	Course c	62.1045	10.82163	36.46307

**Table 2:** Psychometric attributes of college students.

Psychometric attribute description	Meaning for concentrated time period
Person per = (person) has.get(number1);	Code of the input matrix
Name.settext(per.getname());	The additional bias
Objectinputstream in = new objectinputstream();	Channels of physiological signals
Date.settext(per.getdate());	Physiological signal sequences
Frame1.setvisible(true);	The number of frames
Dor.settext(per.getdor());	The number of column vectors
Sex.settext(per.getsex());	Operational data of teachers
Joptionpane.showmessagedialog(null, “”);	Network teaching administrators
New fileinputstream(file)	Use of these temporal information
Phone.settext(per.getphone());	The centralized time period
Person per = (person) enu.nextelement();	The entropy value of a behavior

## Data Availability

The data used to support the findings of this study are available from the corresponding author upon request.
